The article "A Novel Radiomics-Based Machine Learning Framework for Prediction of Acute Kidney Injury-Related Delirium in Patients Who Underwent Cardiovascular Surgery" was published in 2022. Journal: Comput Math Methods Med.

# A Novel Radiomics-Based Machine Learning Framework for Prediction of Acute Kidney Injury-Related Delirium in Patients Who Underwent Cardiovascular Surgery

**DOI:** 10.1155/2022/4242069

**Published:** 2022-03-18

**Authors:** Xin Xue, Wen Chen, Xin Chen

**Affiliations:** ^1^Department of Cardiothoracic Surgery, School of Medicine, Southeast University, Nanjing 210009, China; ^2^Department of Thoracic and Cardiovascular Surgery, Nanjing First Hospital, Nanjing Medical University, Nanjing 210006, China

## Abstract

Acute kidney injury (AKI) can be caused by multiple etiologies and is characterized by a sudden and severe decrease in kidney function. Understanding the independent risk factors associated with the development of AKI and its early detection can refine the risk management and clinical decision-making of high-risk patients after cardiovascular surgery. A retrospective analysis was performed in a single teaching hospital between December 1, 2019, and December 31, 2020. The diagnostic performance of novel biomarkers was assessed using random forest, support vector machine, and multivariate logistic regression. The nomogram from multivariate analysis of risk factors associated with AKI indicated that only LVEF, red blood cell input, and ICUmvat contribute to AKI differentiation and that the difference is statistically significant (*P* < 0.05). Seven radiomics biomarkers were found among 65 patients to be highly correlated with AKI-associated delirium. The importance of the variables was determined using the multilayer perceptron model; fivefold cross-validation was applied to determine the most important delirium risk factors in radiomics of the hippocampus. Finally, we established a radiomics-based machine learning framework to predict AKI-induced delirium in patients who underwent cardiovascular surgery.

## 1. Introduction

Notwithstanding that unprecedented progress has been made in understanding the pathogenesis and development of novel therapeutic strategies, cardiovascular disease remains the leading cause of morbidity and mortality in patients with renal dysfunction, especially acute kidney injury (AKI) [1]. AKI is a complex syndrome caused by multiple etiologies and characterized by a sudden and severe decrease in kidney function, presented with an increase in serum creatinine (SCr) or a reduction in urine output [2, 3]. In a recent study, more than half the patients hospitalized in the intensive care unit (ICU) ward developed AKI [4]. Note that increased AKI severity correlates positively with short- and long-term mortality after discharge [5, 6]. In addition, as established recently, the mortality risk increases significantly with AKI severity, reaching a rate of up to 40–60% [5, 7, 8]. The occurrence rate of AKI might be somewhat affected by differences in socioeconomic statuses [9]. Consequently, the severity of adverse events has become a worldwide medical burden. To the best of our knowledge, regardless of the underlying etiology, there are no effective treatments for AKI once it develops [10]. Clinically, AKI management refers to an early detection of its occurrence for the general critical care population with limited ongoing or recurrent renal injury, consequently providing supportive management of advanced renal dysfunction [11]. Considering the negative impact of AKI on short- and long-term outcomes, it is essential to explore novel methods to identify high-risk patients and diagnose subclinical AKI to improve patient outcomes. As previously described, the development of statistical predictive models for estimating the risk factors of AKI has become possible with the development of clinical informatics and the increasing availability of electronic medical records [12]. Of note, multivariate logistic regression analysis is the most frequently used statistical algorithm to determine risk predictors for the short-term outcome [11]. Several underlying susceptibilities, procedures, or exposures have been identified as risk factors for the occurrence of postoperative AKI, such as older age, chronic kidney disease, comorbidities (e.g., diabetes and hypertension), sepsis, major surgery, and hemodynamic instability [13, 14].

The article "A Novel Radiomics-Based Machine Learning Framework for Prediction of Acute Kidney Injury-Related Delirium in Patients Who Underwent Cardiovascular Surgery" was published in 2022. Journal: Comput Math Methods Med.

An increasing body of evidence has suggested that AKI can significantly affect the brain tissue and function. Ischemic AKI can reportedly cause neuronal pyknosis and an increase in brain microgliomas. In addition, AKI can lead to brain microvascular protein leakage and increased vascular permeability, thereby increasing the risk of cerebrovascular diseases and the incidence of brain dysfunction. The incidence rate of stroke increased significantly with a glomerular filtration rate below 60 ml·min^−1^·1.73 m^−2^ and a Cr/Alb ratio greater than 30 mg/g. Moreover, the United States Renal Disease Database reported that the incidence rate of stroke in uremic people aged >65 years is 9%. The early symptoms in AKI patients with concomitant impaired brain tissue and function include fatigue, apathy, bradykinesia, and an inability to concentrate. In severe cases, delirium, confusion, and coma might occur. In addition, reduced autonomous behavior and slow movement have been documented in animal models of renal ischemia and bilateral nephrectomy.

Acute kidney injury might be associated with numerous brain and hippocampal complications, as it can alter the permeability of the blood–brain barrier. Although the pathogenesis of acute uremic encephalopathy is poorly understood, the potential underlying mechanism contributing to hippocampal involvement includes the release of multiple inflammatory mediators, which lead to hippocampal inflammation and cytotoxicity, neurotransmitter derangement, transcriptional dysregulation, and changes in the expression of apoptotic genes. Impairment of brain function, especially of a structure that has vital activity in learning and memory and is highly sensitive to renal ischemic injury, can ultimately lead to cognitive and functional complications in patients with AKI. Delirium is the most common clinically observed symptom after AKI, as it has a relatively high mortality rate (22%–76%). Liu et al. found that AKI leads to the release of soluble and cellular inflammatory mediators in the brain, which primarily target the hippocampus and increase brain microvascular protein leakage. They also found that severe AKI and bilateral nephrectomy can lead to more pronounced behavior changes than less severe AKI or the combination of sham AKI with surgery and anesthesia [15]. Therefore, early prediction and intervention of hippocampal changes caused by AKI are crucial in reducing patient mortality and improving the prognosis [16].

The article "A Novel Radiomics-Based Machine Learning Framework for Prediction of Acute Kidney Injury-Related Delirium in Patients Who Underwent Cardiovascular Surgery" was published in 2022. Journal: Comput Math Methods Med.

As it is clinically difficult to detect early hippocampal damage, the prognosis is generally poor once the injury occurs, and the associated mortality rate is high. Currently, there is a paucity of efficient and low-cost methods for detecting early hippocampal damage. The current clinical approach involves magnetic resonance imaging (MRI) examination of the hippocampus and qualitative assessment methods to observe morphological changes, with no quantitative analytical methods available. This study is aimed at establishing and validating a machine learning-based quantitative method for noninvasive hippocampal assessment through preoperative cranial computed tomography (CT) instead of magnetic resonance imaging for the early detection of AKI-related hippocampal damage and prompt clinical intervention.

However, early biochemical and clinical data have not been analyzed in studies that sought to predict the risk factors of AKI after surgery [17]. In addition, risk assessment before surgery is crucial to optimize strategies to prevent AKI and AKI-induced hippocampal changes to determine which patients require more intense motorizations after surgery. Overall, the present study seeks to determine the incidence and risk factors of AKI and AKI-associated hippocampal damages in patients who have undergone cardiovascular surgery.

## 2. Materials

### 2.1. Subjects

A retrospective cohort analysis was conducted in a teaching hospital. Patients (age ≥ 18 years) at risk of developing AKI after primary cardiovascular surgery were included in our current study. The exclusion criteria comprised patients with renal insufficiency, acute or chronic kidney disease, or preoperative hemodynamic instability; patients who underwent emergency operation; patients who developed postoperative urinary tract infection or were treated with nephrotoxic drugs or glucocorticoids before or after surgery; and patients without complete clinical data. All patients provided written informed consent before participation. The study was approved by the Medical Ethics Committee of the First Affiliated Hospital of Nanjing Medical University (KY20190404-03-KS-01) and complied with the requirements of the Declaration of Helsinki.

The article "A Novel Radiomics-Based Machine Learning Framework for Prediction of Acute Kidney Injury-Related Delirium in Patients Who Underwent Cardiovascular Surgery" was published in 2022. Journal: Comput Math Methods Med.

### 2.2. AKI Definition and Grouping Design

According to the Kidney Disease Improving Global Outcomes (KDIGO) workgroup [18], the AKI criteria comprise 50% increase in SCr measurements relative to the baseline, SCr increases of more than 0.3 mg/dl within a 48-h interval during 7 days, or urine volume less than 0.5 ml/(kg·h) for 6 h [19]. After cardiovascular surgery, patients who developed postoperative AKI were included in the AKI group, whereas those without AKI were included in the non-AKI group.

### 2.3. Delirium Definition and Grouping Design

According to the DSM-IV-TR criterion [20], the diagnostic criteria for delirium included the following: (A) disturbance of consciousness (i.e., reduced clarity of environmental awareness) with reduced ability to focus, sustain, or shift attention. (B) A change in cognition or the development of a perceptual disturbance that is not better accounted for by a preexisting, established, or evolving dementia. Other common features of delirium include sleep disorders (such as changes in sleep–wake cycles), changes in psychomotor activity, and abnormal neurobehavioral symptoms. Delirium cases were divided into hyperactive type (HT), inhibited type (IT), and mixed type (MT). Patients with HT presented with a state of restlessness and high alertness to the surrounding environment. Patients with IT exhibited poor arousal, lethargy, and weakness. Because this type of delirium is nondestructive, the symptoms are usually undetectable. Patients expressing both phenotypes were classified as MT. Within 48 h of cardiovascular surgery, the included patients were examined by psychologists and classified using the abovementioned criteria.

## 3. Methods

### 3.1. Clinical Data Collection

Three hundred and twenty patients who underwent cardiovascular surgery from December 1, 2019, to December 31, 2020, were retrieved from hospital's electronic medical records. Finally, 227 patients were included in our study and separated into training and validation groups. The preoperative data mainly included demographic characteristics (age, gender), height, body weight, body mass index, smoking and drinking history, comorbidities (hypertension, diabetes, and cardiovascular disease), central venous pressure, left ventricular ejection fraction (LVEF), coronary arteriography, and clinical laboratory data (hemoglobin, albumin, hematocrit, baseline SCr, N-terminal pro-brain natriuretic peptide (NT-proBNP), neutrophil gelatinase-associated lipocalin (NGAL), fatty acid-binding protein (FABP), troponin I (TnI), and blood glucose). The intraoperative data comprised the cardiopulmonary bypass (CPB) time, type of surgery, extracorporeal circulation urine output, ultrafiltration volume, and red blood cell input (RBCI) on the surgery day. Finally, the postoperative data included the length of ICU stay, mechanical ventilation auxiliary time (MVAT), and continuous renal replacement therapy (CRRT) use.

The article "A Novel Radiomics-Based Machine Learning Framework for Prediction of Acute Kidney Injury-Related Delirium in Patients Who Underwent Cardiovascular Surgery" was published in 2022. Journal: Comput Math Methods Med.

### 3.2. Imaging Data Collection

All patients underwent brain CT before cardiovascular surgery; CT images with an axial slice thickness of 1 mm were retrospectively collected between December 1, 2019 and December 31, 2020. All study subjects were older than 18 years, and a normal hippocampus was confirmed before surgery.  Figure 1 demonstrates the machine learning process adopted in the study and patient data distribution.

### 3.3. Image Preprocessing and Hippocampus Autosegmentation

After the brain CT images were obtained, a deep learning method was applied to generate a visual MRI image set for hippocampus auto-segmentation, as reported by Li et al. [21]. The traditional CT image and artificial intelligence brain library were used to reconstruct the MRI image from the virtual image library closest to the patient's brain anatomy and to perform CT-MR image fusion through artificial intelligence methods. Accordingly, a virtual MRI could determine the location of the hippocampus from the CT image and delineate it. In addition, bias field correction was applied for virtual MRI image noise reduction and preprocessing. Regions of interest (ROIs) were used as the range for feature extraction of the hippocampus. To compensate for the effect of variable voxel size on image analysis, all CT images were resampled to pixel dimensions of 1 mm × 1 mm × 5 mm. To reduce the errors associated with manual delineation of the hippocampus and improve the delineation efficiency, a rigorously tested and internally developed delineation program based on artificial intelligence was used to delineate the hippocampus before and after the cardiovascular surgery. As enhanced CT is not routinely used in clinical practice, cases with only plain CT scans were also collected to delineate the hippocampus. According to the literature, the two images exhibit no statistical significance in delineating the volume and boundary of the hippocampus. The mean Dice similarity coefficient and average Hausdorff distance of the two image sequences were 0.90 and 1.6 mm, respectively. All above steps are explained in Figure 2, the process of automatically delineating the hippocampus ROI from CT and radiomics feature extraction.

The article "A Novel Radiomics-Based Machine Learning Framework for Prediction of Acute Kidney Injury-Related Delirium in Patients Who Underwent Cardiovascular Surgery" was published in 2022. Journal: Comput Math Methods Med.

### 3.4. Image Feature Extraction

Quantitative radiomics analysis was conducted on the hippocampus region. A total of 661 radiomics features characterizing the intensity and texture of the hippocampus were extracted. Wavelet transformation was performed on the hippocampus region to quantify the hippocampus in multiple dimensions.

The intensity features measured the gray-level distribution in the tumor region and quantified in terms of mean, energy, entropy, variance, skewness, and kurtosis. The texture features that characterized the tumor texture properties were based on the gray-level cooccurrence matrix (GLCM), gray-level size-zone matrix (GLSZM), gray-level run-length matrix (GLRLM), and neighborhood gray-tone-difference matrix (NGTDM), including homogeneity (GLCM), small-zone emphasis (GLSZM), short-run emphasis (GLRLM), and complexity (NGTDM). Details of the texture features, including the category and feature names, are provided in Table 1.

Wavelet selection was performed by selecting the high-frequency parts (H) or low-frequency parts (L) of the wavelet components of the tumor region at the very axis. Eight categories of wavelet features were acquired and labeled as HHH, HHL, HLH, LHH, LLL, LLH, LHL, and HLL. The HLH category features comprised texture features derived from the tumor region after high-frequency wavelet selection on the *x*-axis and *z*-axis and low-frequency wavelet selection on the *y*-axis.

### 3.5. Image/Clinical Feature Selection

To compensate for the accuracy of AD on hippocampus delineation, the texture analysis method was repeated two more times by performing morphological erosion and expansion of all pixels on the initial contour of the ROI. Only radiomics features that showed a high correlation (>0.99) with the erosion and expansion of the ROI were used for further analysis.

Specific feature screening steps:

1. After feature extraction, the null features were removed, and features that had no omics feature changes before and after the operation were deleted, leaving 714 features
2. The MWU test was conducted to delete features unrelated to the result variable (*n* = 103), and 611 features were left. The study samples were divided into two groups (delirium and no delirium) according to our data. The Mann–Whitney *U*-test/Wilcoxon rank-sum test was used to compare the preoperative and postoperative hippocampal radiomics characteristics of different groups. The characteristics that exhibited significant differences between the groups were screened. The MWU test excluded 107 features that exhibited no statistical differences within the group (FDR was used to obtain corrected *P* values).
3. Variance/standard deviation analysis: the features whose standard deviation (SD) was less than 0.05 were deleted, resulting in 490 features
4. Correlation detection: redundant features with a Pearson correlation index ≥ 0.99 were deleted, and features highly correlated with the classification results were retained. The number of feature variables was reduced from 491 to 163
5. Finally, LASSO dimensionality reduction was performed, features were reduced from 163 to 7, and the smallest MSE was selected. As a result, the simplest predictive classification model obtained with one SD consisted of only eight variables

The article "A Novel Radiomics-Based Machine Learning Framework for Prediction of Acute Kidney Injury-Related Delirium in Patients Who Underwent Cardiovascular Surgery" was published in 2022. Journal: Comput Math Methods Med.

### 3.6. Image/Clinical Signature Construction

A radiomics signature and a clinical signature were built by summing the features multiplied by their coefficients. The prediction value of integration of radiomics and clinical features was tested using a multivariable logistic regression model. Finally, the prediction model's performance was assessed by calculating the AUC of the ROCs.

### 3.7. Image/Clinical Signature Validation

The signatures were established using a fourfold cross-validation approach. The patients were randomly separated into five folds. Three out of the four folds were used for feature selection at a *λ* value. The resulting signature was then tested on the other fold patients. The binomial deviance of fivefold cross-validation was used to select the best *λ* value for the least binomial deviance.

### 3.8. Statistical Analysis

Measured data were expressed as absolute numbers and percentages or mean ± standard deviation ($\overset{®}{x}\pm s$) and interquartile ranges (25th and 75th percentiles) when applicable. Continuous variables were compared using the Mann–Whitney *U* test, and categorical variables were compared using the chi-square or Fisher's exact test. All calculations were performed using SPSS 22.0 Statistical Software (SPSS, Inc., Chicago, IL, USA) and MedCalc Statistical Sofware, version 19.0.4 (MedCalc Software bvba, Ostend, Belgium). Univariate logistic regression was conducted to screen potential risk factors significantly associated with AKI. The multivariate logistic regression analysis included factors that exhibited statistical significance during univariate analysis (*P* value < 0.05) to stratify postoperative AKI-related risk factors. The stepwise forward method was used for variable selection. Measures of effect were reported using odds ratios for both crude and adjusted analysis, followed by a 95% confidence interval, and a *P* value < 0.05 was used to determine statistical significance. Furthermore, the diagnostic performance of novel biomarkers was assessed by calculating the areas under the receiver-operator characteristic curves (AUC); pairwise comparison of ROC curves was performed for AKI risk and AKI-associated hippocampal changes and delirium.

The article "A Novel Radiomics-Based Machine Learning Framework for Prediction of Acute Kidney Injury-Related Delirium in Patients Who Underwent Cardiovascular Surgery" was published in 2022. Journal: Comput Math Methods Med.

## 4. Experimental Results and Discussion

### 4.1. Characteristics and Outcomes of Patients

Between December 1, 2019, and December 31, 2020, 320 patients were at risk of developing AKI in the cardiothoracic surgery department, and 227 patients were involved in the final study cohort. A flowchart of our study is provided in Figure 3. According to the KDIGO clinical practice guidelines, 66 patients were diagnosed with hospital-acquired AKI within a week after the cardiovascular surgery, of which 29 patients (43.94%) exhibited hippocampal changes and delirium. Surgical procedures in the AKI group included coronary artery bypass surgery (*n* = 19), valve replacement (*n* = 29), and a combination of two or more cardiovascular surgical operations (*n* = 18). Surgical procedures in the non-AKI group also included coronary artery bypass surgery (*n* = 38), valve replacement (*n* = 103), and a combination of two or more cardiovascular surgical operations (*n* = 20). At the end of the study, two patients who required CRRT after valve replacement surgery or coronary artery bypass surgery survived. Of the four patients (1.76%) who died, three developed postoperative AKI, and the mortality rate in the AKI group was higher than that in the non-AKI group (*P* ≤ 0.01). Detailed patient characteristics grouped according to the KDIGO workgroup are provided in Table 1. Detailed patient characteristics with and without delirium are provided in Table 2.

### 4.2. Univariate Logistic Regression Analyses of Risk Factors for AKI

Upon admission, the older patients, especially those older than 60 years, harbored a higher risk of AKI. As shown in Table 1, patients with preexisting complications were prone to AKI, such as diabetes. Patients with anemia were at an increased risk of AKI, especially those with low serum albumin levels. Conversely, no significant correlation was found between the other demographic and physiological variables in AKI patients (*P*_s_ > 0.05). To increase the diagnostic accuracy, novel biomarkers, including NGAL, TnI, FABP, and NT-proBNP, were also investigated in this setting. Univariate analysis revealed that the urinary NGAL level was higher in patients with AKI than those without (*P* < 0.05). In contrast, there were no significant differences among the serum levels of TnI, FABP, and NT-proBNP between patients with and without AKI. Additionally, there was no remarkable difference in the coronary angiography findings between patients with and without AKI (*P* > 0.05).

The article "A Novel Radiomics-Based Machine Learning Framework for Prediction of Acute Kidney Injury-Related Delirium in Patients Who Underwent Cardiovascular Surgery" was published in 2022. Journal: Comput Math Methods Med.

Analysis of routinely used intraoperative variables showed that an increased risk of AKI was associated with a combination of surgical operations, prolonged CPB therapy, longer duration of surgery, or erythrocyte transfusions on the day of surgery. Conversely, there were no significant differences in other intraoperative variables between patients with and without AKI, such as interval, aortic occlusion time, urine output, and ultrafiltration volume (*P*_s_ > 0.05). Notably, postoperative AKI was associated with worse outcomes, such as prolonged mechanical ventilation auxiliary time, length of ICU stay, and hospitalization time.

### 4.3. Diagnostic Performance of Novel Biomarkers Using Random Forest, Support Vector Machine, and Multivariate Logistic Regression

When EF, RBCI, and ICUmvat were entered in the regression equation, ICUmvat had the largest impact on the entire model, followed by EF and RBCI. We assumed that when ICUmvat was equal to 60 h, EF was 40%, and RBCI was 4, yielding scores of 30, 50, and 25, respectively (the red arrow in Figure 4), and a total score of 105. A total score greater than 70% was obtained for the predicted risk of AKI using the above three variables. This approach is simple and can be easily implemented in clinical practice.

Figure 4 demonstrates the nomogram obtained from multivariate log regression analysis of risk factors associated with AKI, including EF, RBCI, and ICUmvat. We created a nomogram with these three variables for easy implementation during clinical practice. Meanwhile, the diagnostic performance of novel biomarkers EF, RBCI, and ICUmvat, and the clinical signature was assessed using ROC curves (Figure 5).

Prediction of AKI and AKI-related hippocampus changes after the cardiovascular surgery is demonstrated in Table 3. The AUC scores of the fivefold cross-validation after the application of multiple logistic regression, random forest, and support vector machine are summarized in Tables 4 and 5 (Figure 6) and Table 6 (Figure 7), respectively. The SVM model that performed the best during the fivefold cross-validation could distinguish AKI from non-AKI, as demonstrated in the heat map (Figure 8).

The article "A Novel Radiomics-Based Machine Learning Framework for Prediction of Acute Kidney Injury-Related Delirium in Patients Who Underwent Cardiovascular Surgery" was published in 2022. Journal: Comput Math Methods Med.

The “cmdscale” function can implement traditional multidimensional scaling, also known as principal coordinate analysis. It takes the interior point distance matrix as the input and outputs a series of points. Ideally, these points are two-dimensional or three-dimensional. The Euclidean distance between them produces the same distance matrix as the original; accordingly, the scatter plot of these points can objectively present the original distance.

### 4.4. Multilayer Perceptron-Based Prediction Model Establishment for AKI-Led Delirium

Before developing the predictive model, the collected data were randomly divided into training (70%) and validation (30%) datasets. The training dataset was used to construct predictive models using machine learning algorithms (multilayer perceptron (MLP) was mainly used here). Fivefold cross-validation was used to continuously adjust model's parameters to reduce the chance of overfitting and then verify and compare the final performance of each model in the validation dataset. AUC, sensitivity, specificity, and accuracy were used to compare different models. For modeling and statistical analysis, the Rstudio neural network package version 1.44.2 (https://cran.r-project.org/web/packages/neuralnet/index.html) and Python programming software version 3.9 (Python software, http://www.python.org/) were used. An MLP network with two hidden layers was built using the training dataset. Each hidden layer contained 11 neurons. The same network structure was used for the validation dataset, but the training weight parameters of each neuron were obtained after optimizing the training dataset. The softmax activation function was used in the final output layer before the network could output the final results.

Seven radiomics biomarkers were found in 65 patients to be highly correlated with AKI-related delirium (Table 7).

The importance of the variables was determined using the MLP model (Figure 9); fivefold MLP training and validation was applied to determine the most important delirium risk factors in the radiomics of the hippocampus. The MLP network structure and model performance are presented in Figures 10 and 11, respectively.

### 4.5. Discussion

Cardiac surgery-associated acute kidney injury (CSA-AKI) is a well-documented complication following cardiac surgery, associated with increased morbidity and mortality, prolonged hospital stay, and higher medical costs [22]. Much heterogeneity surrounds AKI incidence after cardiovascular surgery due to the differences in research objects, research methods, AKI definitions, diagnosis and treatment levels of medical centers, and selected models. Based on the KDIGO clinical practice guidelines, 66 patients in our present study were diagnosed with hospital-acquired AKI within a week after cardiovascular surgery, with an incidence rate of 29.07% (range 5%–30%), consistent with the literature [23, 24]. To appropriately manage CSA-AKI, a precise prediction model for identifying high-risk patients is required to optimize the postoperative treatment strategy.

The article "A Novel Radiomics-Based Machine Learning Framework for Prediction of Acute Kidney Injury-Related Delirium in Patients Who Underwent Cardiovascular Surgery" was published in 2022. Journal: Comput Math Methods Med.

To analyze numerous variables with nonlinearity and complex relationships associated with CSA-AKI development, an alternative and effective approach is required to develop precise prediction models. Over the years, machine learning has been applied in different areas of medicine, such as outcome prediction, diagnosis, medical image interpretation, and treatment [25, 26]. The advantage of this completely data-driven learning without reliance on rule-based programming is that machine learning constitutes a reasonable approach. Accordingly, in the present study, machine learning methods especially in predictive control techniques were applied to develop a model for the accurate prediction of CSA-AKI [27].

Previous studies have addressed the relationship between cardiac dysfunction and AKI risk in various clinical settings. For instance, in patients who underwent coronary artery bypass grafting and had preserved systolic function, preoperative *E*/*e*′ > 15 was a strong independent predictor of AKI [28]. Moreover, among patients who underwent primary coronary intervention due to ST-segment elevation myocardial infarction, a high *E*/*e*′ ratio was associated with an increased risk of AKI [29]. Another study showed that decreased LVEF was associated with a faster deterioration of the renal function [30]. Patients with heart failure who underwent coronary artery bypass surgery exhibited an increased risk for AKI postoperatively, even after adjustment for comorbidities, such as LVEF. Among patients with heart failure, having a severely reduced LVEF was associated with AKI more than those with preserved LVEF [31]. The present study also supported these previous results. In addition, the present study showed that systolic and diastolic heart dysfunction, characterized by LVEF differences, was associated with AKI development in hospitalized patients. Therefore, echocardiographic monitoring of heart dysfunction can be added to the prediction models of AKI and possibly to real clinical practice to identify high-risk patients and improve outcomes.

Meanwhile, anemia has been reported as a potential modifiable risk factor for postoperative AKI [32, 33]. Anemia is associated with an increased AKI risk, mainly in the surgical setting [33]. However, preoperative anemia is associated with an increase in the probability of erythrocyte transfusion, risk of postoperative renal failure, and mortality, as more intraoperative blood transfusion implies more postoperative bleeding [34]. Accumulating evidence has demonstrated a dose-dependent association between the volume of red blood cells (RBCs) and AKI severity [35, 36]. Consistent with the literature, we found that erythrocyte transfusions on the surgery day were associated with an increased rate of AKI. A series of changes that RBCs experience during storage, including decreased deformability, increased fragility, progressive hemolysis, and accumulation of free hemoglobin and iron, have been proposed as mechanisms responsible for transfusion-associated AKI [37].

The article "A Novel Radiomics-Based Machine Learning Framework for Prediction of Acute Kidney Injury-Related Delirium in Patients Who Underwent Cardiovascular Surgery" was published in 2022. Journal: Comput Math Methods Med.

In addition, our analysis of intraoperative variables demonstrated that adult patients had a high incidence of AKI after CPB heart surgery and required a prolonged length of ICU or hospital stay; severe AKI could increase perioperative mortality by 3–8 times [38]. An increasing body of evidence has suggested that postoperative AKI occurrence is associated with short-term adverse outcomes [39, 40]. The present study showed that patients who developed AKI required invasive mechanical ventilation, higher mortality, prolonged length of ICU stay, and longer hospitalization time. Exposure to surgery and nephrotoxins is one of the specific modifiable factors, subsequently contributing to AKI development [5, 18, 41]. Additionally, AKI has been associated with increased in-hospital mortality and short- and long-term mortalities after discharge [6]. It has previously been reported that the long-term prognosis is still poor for AKI patients, even with complete recovery of the renal function [42]. Accordingly, it is important to explore the risk factors associated with short- and long-term outcomes of AKI patients.

As shown in Figure 5, the multivariate logistic regression method showed that the predictive performance of a single clinical or laboratory index for AKI was limited. The largest and smallest AUC values were found for RBCI (0.651) and ICUmvat (0.559), respectively, suggesting that although these indicators are effective in predicting AKI and are statistically significant during logistic regression, their predictive power is largely limited. However, the predictive performance was significantly enhanced when the three variables were integrated into a prediction model (AUC value 0.753). In addition, although the random forest-based prediction model yielded excellent performance in the training set, the AUC values ranged from 0.881 to 1 during training of the fivefold cross-validation model. However, in the subsequent validation dataset, the model's generalization ability was average, and the maximum AUC was only 0.714. This finding shows that the random forest model exhibits transitional fitting in the training set. The above findings suggest that the generalization of our model was average, with a lower performance yield than the multivariate logistic regression method. This observation is related to settings such as the number of random forest trees during the design of the random forest model. Pruning and pruning settings have always been challenging in machine learning, requiring constant trial and error to balance the training and validation datasets. The support vector machine-based model performed better than the above two methods, with an AUC value of 0.812 for the best model. When the simple neural network of MLP was used to predict the probability of delirium caused by AKI, although the number of hidden layers was 2 and the number of neurons in each layer was 10, the machine learning MLP model yielded excellent performance in the training and validation datasets. The average AUC reached 0.903, suggesting that our simple neural network is efficient for the two-class prediction models and yields excellent prediction results with a simpler network structure.

The article "A Novel Radiomics-Based Machine Learning Framework for Prediction of Acute Kidney Injury-Related Delirium in Patients Who Underwent Cardiovascular Surgery" was published in 2022. Journal: Comput Math Methods Med.

This study has some limitations. Our analysis used only single-center data, with a relatively small sample size. The performance of the machine learning algorithm might differ when applied to larger datasets with heterogeneous patient characteristics. As such, external validation is required to prevent overfitting. Future prospective studies are required to evaluate the application of machine learning-based predictive models during clinical practice to identify patients at high risk of AKI and improve outcomes.

## 5. Conclusion

Because of the high incidence of AKI, understanding the independent risk factors associated with the development of AKI and its early detection is helpful in the risk management and clinical decision-making of high-risk patients after cardiovascular surgery. A radiomics-based machine learning framework can predict AKI-related delirium in patients who have undergone cardiovascular surgery.

## Figures and Tables

**Figure 1:** Machine learning analysis process of AKI and AKI-led delirium on clinical and CT radiomics parameters.

**Figure 2:** The process of automatically delineating the hippocampus ROI from CT and radiomics feature extraction.

**Figure 3:** Flow chart representing the patient selection process and groups.

**Figure 4:** Nomogram from multivariate analysis of risk factors associated with AKI.

**Figure 5:** Diagnostic performance of novel biomarkers using receiver-operative characteristic curves of EF, RBCI, ICU_mvat_, and clinical signature. (a–d) stands for the performance of novel biomarkers of EF, RBCI, ICUmvat, and clinical signature, respectively.

The article "A Novel Radiomics-Based Machine Learning Framework for Prediction of Acute Kidney Injury-Related Delirium in Patients Who Underwent Cardiovascular Surgery" was published in 2022. Journal: Comput Math Methods Med.

**Figure 6:** ROC curve of the 5 folds in training and testing sets and the best performance Signature of random forest (RF) model. The first row (a–e) represents the ROC calculated by 5 folds of the training set; the second row (f–j) represents the ROC calculated for 5 folds of the test set.

**Figure 7:** (a) The ROC curve of the best performance signature of SVM model, (b) which reflects the multidimensional scale transformation diagram of AKI and non-AKI.

**Figure 8:** Heat map of the best performance signature of SVM model with the horizontal axis represents samples, and the vertical axis represents different predictors.

**Figure 9:** The importance of the variables determined by the MLP model; a 5-fold MLP training and testing was applied to determine the most important delirium risk factors in radiomics of the hippocampus.

**Figure 10:** The MLP training network structure which includes two hidden layer.

**Figure 11:** Prediction model compared MLP model performance in training, testing, and validation set with the best SVM model.

**Table 1:** Characteristics of patients of risk factors associated with AKI after cardiovascular surgery (*N* = 227).

Variables	AKI group (*n* = 66)	Non-AKI group (*n* = 161)	*χ* ^2^/*F*/*t*/*Z*	*P* value
Demographic				
Gender (male) (*n* [%])	39 (59.09)	82 (50.93)	1.293	0.256
Age ≥ 60 (year)	44 (66.67)	84 (52.17)	4.669	0.031
Height (cm) ($\overset{®}{x}\pm s$)	164.12 ± 9.64	163.52 ± 8.63	0.477	0.634
Weight (kg) ($\overset{®}{x}\pm s$)	66.89 ± 11.51	66.69 ± 10.71	0.988	0.323
BMI (kg/m^2^) ($\overset{®}{x}\pm s$)	1.797 ± 0.178	1.793 ± 0.169	0.146	0.884
Smoking history (*n* [%])	17 (25.75)	28 (17.39)	2.400	0.121
Drinking history (*n* [%])	8 (12.12)	9 (5.59)	2.198	0.138
Laboratory				
Hematocrit ($\overset{®}{x}\pm s$) (%)	24.92 ± 3.89	25.08 ± 3.80	-1.425	0.155
Albumin (g/l) ($\overset{®}{x}\pm s$)	38.25 ± 3.36	40.12 ± 3.40	-3.794	0.000
NGAL (ng/ml) (*M* [IQR])	82.3 (51.7, 153.7)	49.2 (34.9, 117.2)	-3.272	0.001
TnI (>0.5 ng/ml) (*n* [%])	12 (18.18)	24 (14.90)	0.327	0.568
FABP (>2.5 ng/ml) (*n* [%])	17 (25.75)	37 (22.98)	0.243	0.622
NT-prBNP (>300 pg/ml) (*n* [%])	20 (30.30)	24 (14.91)	2.079	0.149
Coronary angiography (*n* [%])	49 (74.24)	112 (69.56)	0.397	0.529
Clinical				
Hypertension (*n* [%])	33 (50.00)	76 (47.20)	0.180	0.671
Diabetes (*n* [%])	25 (37.88)	28 (17.39)	10.979	0.001
Anemia (*n* [%])∗	25 (37.87)	20 (12.42)	19.086	0.000
LVEF ($\overset{®}{x}\pm s$) (%)	58.43 ± 7.42	60.42 ± 5.39	-1.807	0.024
CVP (cmH_2_O) ($\overset{®}{x}\pm s$)	9.076 ± 3.400	8.621 ± 2.629	0.973	0.333
Type of surgery (*n* [%])			9.900	0.007
Coronary artery bypass surgery	19 (28.79)	38 (23.60)		
Valvuloplasty	29 (43.94)	103 (63.98)		
Combined surgery∗∗	18 (27.27)	20 (12.42)		
CPB time (>120 minutes) (*n* [%])	34 (51.52)	45 (27.95)	11.456	0.001
Duration of surgery (>6 hours) (*n* [%])	40 (60.60)	69 (42.85)	5.908	0.015
Aortic occlusion time (minute) (*M* [IQR])	108 (83.5, 140.5)	97 (82.0, 129.0)	-1.670	0.095
Red blood cell input (*n* [%])	23 (34.85)	10 (6.21)	30.899	0.000
Urine output (ml) (*M* [IQR])	200 (100, 300)	200 (150, 350)	-1.619	0.105
Ultrafiltration volume (ml) (*M* [IQR])	1350 (800, 2250)	1500 (800, 2070)	-0.720	0.472
ICU length of stay (day) (*M* [IQR])	2 (1, 4)	1 (1, 2)	-5.4189	0.000
Mechanical ventilation time (hour) (*M* [IQR])	14 (10.0, 20.25)	11 (7.5, 14.0)	-3.822	0.000
CRRT (*n* [%])	2 (3.0)	0 (0.00)	Fisher's	0.246
Hospitalization time (day) ($\overset{®}{x}\pm s$)	18.70 ± 5.52	15.78 ± 5.61	3.591	0.000

Notes: ∗Preoperative anemia was defined as a hemoglobin less than 110 g/l in female patients and 120 g/l in male patients; ∗∗Combined surgery was referred to a combination of two or more surgical operations. Abbreviations: BMI: body mass index; CPB: cardiopulmonary bypass; CVP: central venous pressure; CRRT: continuous renal replacement therapy; FABP: fatty acid-binding protein; IABP: intra-aortic balloon pump; ICU: intensive care unit; LVEF: left ventricular ejection fraction; *M* [IQR]: median [inter quartile range]; NGAL: neutrophil gelatinase-associated lipocalin; NT-prBNP: N-terminal probrain natriuretic peptide; TnI: troponin I.

The article "A Novel Radiomics-Based Machine Learning Framework for Prediction of Acute Kidney Injury-Related Delirium in Patients Who Underwent Cardiovascular Surgery" was published in 2022. Journal: Comput Math Methods Med.

**Table 2:** Characteristics of patients with delirium and without delirium (*N* = 66).

	Delirium group (*N* = 29)		Nondelirium group (*N* = 36)			
	Average	sd	Average	sd	*P* value	*q* value
Age	62.364	11.054	62.097	11.214	0.543	0.283
Weight	64.927	9.093	64.758	9.845	0.784	0.682
Height	165.200	8.322	164.661	9.009	1.231	1.231
BMI	1.803	0.144	1.798	0.158	0.068	0.015
Hemoglobin	131.291	21.513	131.468	22.320	0.342	0.149
Hematocrit	25.182	3.087	24.710	3.400	0.743	0.614
Albumin	39.485	3.285	39.349	3.455	0.066	0.011
NGAL	130.778	67.210	130.911	66.236	0.593	0.361
TnI	0.348	0.836	0.479	1.606	0.055	0.005
FABP	1.580	2.959	1.721	3.103	0.784	0.716
NT-prBNP	376.628	501.617	408.349	568.687	0.124	0.038
LVEF	62.273	5.182	61.565	6.385	0.112	0.029
CVP	8.618	3.670	8.548	3.640	0.054	0.002
Type of surgery	2.164	1.290	2.129	1.263	0.342	0.164
CPB time	112.255	36.932	115.258	38.488	0.674	0.527
RBCI	0.487	1.527	0.529	1.524	0.634	0.413
Aortic occlusion time	73.155	28.342	76.218	29.587	0.894	0.855
Ultrafiltration volume	1820.982	1096.451	1858.935	1121.492	0.556	0.314
ICU length of stay	1.927	2.641	2.290	3.050	0.064	0.008
ICU mechanical ventilation time	12.825	13.227	14.974	17.253	0.321	0.126
Hospitalization time	17.576	8.069	18.237	7.965	0.667	0.493

The article "A Novel Radiomics-Based Machine Learning Framework for Prediction of Acute Kidney Injury-Related Delirium in Patients Who Underwent Cardiovascular Surgery" was published in 2022. Journal: Comput Math Methods Med.

**Table 3:** Multivariate analysis of risk factors associated with AKI after cardiovascular surgery.

	Coefficients	St. error	*Z*	*P* value
Intercept	0.0738	2.4390	0.0300	0.9759
Diabetes	0.2187	0.1543	1.4170	0.1563
NGAL	0.0004	0.0007	0.4870	0.6260
TnI	-0.1471	0.1273	-1.1550	0.2480
Albumin	-0.0265	0.0527	-0.5030	0.6146
LVEF	-0.0420	0.0209	-2.0060	0.0449∗
CPB time	-0.0001	0.0085	-0.0110	0.9912
Aortic occlusion time	0.0173	0.0109	1.5820	0.1137
RBCI	0.2451	0.1346	1.8210	0.0485∗
Ultrafiltration capacity	0.0001	0.0002	0.6930	0.4882
ICUmvat	0.0195	0.0089	2.1920	0.0284∗
Cleveland	0.2304	0.1421	1.6210	0.1050

Abbreviations: 95% CI: 95% confidence interval; CPB: cardiopulmonary bypass; ICU: intensive care unit; NGAL: neutrophil gelatinase-associated lipocalin; OR: odds ratio; SE: standard error. ^∗^*P* value < 0.05.

**Table 4:** 5-fold cross-validation results of AUC after multiple logistic regression (MLR).

Signature	AUC	Precision	Recall	*F*-score	Accuracy	Delong test for AUC values
Training set						
Fold-1	0.633	0.696	0.320	0.438	0.773	*Z* = 8.551, *P* ≤ 0.01
Fold-2	0.594	0.619	0.250	0.356	0.739	
Fold-3	0.635	0.667	0.340	0.450	0.757	
Fold-4	0.640	0.708	0.333	0.453	0.773	
Fold-5	0.662	0.639	0.426	0.511	0.757	
Average	0.633	0.666	0.334	0.442	0.760	
Testing set						
Fold-1	0.596	0.200	0.500	0.286	0.667	*Z* = 6.321, *P* ≤ 0.01
Fold-2∗	0.817	0.385	0.833	0.526	0.804	
Fold-3	0.745	0.583	0.636	0.609	0.800	
Fold-4	0.609	0.214	0.500	0.300	0.689	
Fold-5	0.503	0.182	0.250	0.211	0.667	
Average	0.654	0.313	0.544	0.386	0.725	
Best model in validation set∗	AUC	Precision	Recall	*F*-score	Accuracy	
	0.753	0.667	0.277	0.391	0.934	

**Table 5:** AKI classification performance using clinical-based random forest (RF) model.

Signature	AUC	Precision	Recall	*F*-score	Accuracy	Delong test for AUC values
Training set						
Fold-1	0.957	0.714	0.909	0.800	0.889	*Z* = 11.203, *P* ≤ 0.01
Fold-2	0.934	1.000	0.308	0.471	0.800	
Fold-3	0.927	1.000	0.636	0.778	0.909	
Fold-4	0.881	1.000	0.462	0.632	0.848	
Fold-5	1.000	1.000	1.000	1.000	1.000	
Average	0.940	0.943	0.663	0.736	0.889	
Testing set						
Fold-1	0.686	0.471	0.296	0.364	0.691	*Z* = 9.674, *P* ≤ 0.01
Fold-2	0.665	0.522	0.231	0.320	0.718	
Fold-3	0.583	0.267	0.074	0.116	0.665	
Fold-4	0.659	0.485	0.308	0.376	0.706	
Fold-5∗	0.714	0.571	0.500	0.533	0.767	
Average	0.661	0.463	0.282	0.342	0.709	
Best model in validation set∗	AUC	Precision	Recall	*F*-score	Accuracy	Delong test for AUC values
	0.817	0.620	0.677	0.647	0.788	

**Table 6:** The AKI classification performance using clinical-based support vector machine (SVM) model.

Signature	AUC	Precision	Recall	*F*-score	Accuracy	Delong test for AUC values
Testing set						
Fold-1	0.535	0.973	0.777	0.864	0.729	*Z* = 2.551, *P* = 0.042
Fold-2	0.500	1.000	0.767	0.868	0.696	
Fold-3	0.558	0.861	0.786	0.822	0.700	
Fold-4	0.548	0.938	0.777	0.850	0.724	
Fold-5	0.500	1.000	0.777	0.874	0.713	
Average	0.528	0.954	0.777	0.856	0.712	
Training set						
Fold-1	0.612	0.247	1.000	0.396	0.124	*Z* = 5.551, *P* = 0.019
Fold-2	0.769	0.865	0.776	0.818	0.867	
Fold-3	0.650	0.938	0.818	0.874	0.844	
Fold-4	0.808	0.849	0.776	0.811	0.889	
Fold-5∗	0.615	0.938	0.776	0.849	0.778	
Average	0.731	0.882	0.778	0.826	0.849	
Best model in validation set∗	AUC	Precision	Recall	*F*-score	Accuracy	Delong test for AUC values
	0.812	0.821	0.742	0.780	0.870	

The article "A Novel Radiomics-Based Machine Learning Framework for Prediction of Acute Kidney Injury-Related Delirium in Patients Who Underwent Cardiovascular Surgery" was published in 2022. Journal: Comput Math Methods Med.

**Table 7:** Radiomics biomarker correction with AKI-led delirium.

	Delirium	
	OR	95% CI
GLCM∗315.4ClusterProminence	1.45	0.98-1.89
GLCM270.7Contrast	2.33	1.76-2.97
GLCM333.7InverseVariance	1.56	1.11-1.98
GLCM180.7Energy	2.67	2.03-3.19
GLCM225.1InformationMeasureCorr1	1.97	0.98-2.23
GLCM225.4Correlation	1.19	0.87-1.34
GLCM315.4Correlation	2.54	1.78-3.07

Notes: ∗GLCM: gray level cooccurrence matrices.

## Data Availability

Data are available on request from the authors due to ethical restrictions of our patients' privacy.
